# 23G Minimally Invasive Vitrectomy Combined with Glaucoma Drainage Valve Implantation and Phacoemulsification Cataract Extraction for Neovascular Glaucoma Secondary to Proliferative Diabetic Retinopathy with Vitreous Hemorrhage

This article has been retracted.

**DOI:** 10.1155/2022/7393661

**Published:** 2022-08-04

**Authors:** XiaoLing Shi, Nuo Dong, Yuanyuan Liang, Lin Zheng, Xiaobo Wang

**Affiliations:** ^1^Eye Institute and Affiliated Xiamen Eye Center of Xiamen University, School of Medicine, Xiamen University, Xiamen, 361100 Fujian, China; ^2^Fujian Provincial Key Laboratory of Corneal & Ocular Surface Diseases, Xiamen, 361002 Fujian, China; ^3^Department of Ophthalmology, Affiliated People's Hospital & Zhenjiang Kangfu Eye Hospital, Jiangsu University, Zhenjiang, 212003 Jiangsu, China; ^4^Huaihe Hospital of Henan University, Kaifeng, 475000 Henan, China

## Abstract

**Objective:**

To evaluate the clinical efficacy of the combined application of 23G minimally invasive vitrectomy, glaucoma drainage valve implantation, and phacoemulsification cataract extraction in the treatment of neovascular glaucoma (NVG) secondary to proliferative diabetic retinopathy (PDR) combined with vitreous hemorrhage (VH).

**Methods:**

Eighty-three patients (91 eyes) with PDR diagnosed as NVG phase III complicated with VH from June 2018 to May 2020 were selected as the study subjects. The subjects were randomly divided into 3 groups: group A was treated with 23G minimally invasive vitrectomy combined with glaucoma drainage valve implantation; group B was given 23G minimally invasive vitrectomy combined with phacoemulsification cataract extraction; and group C was treated with 23G minimally invasive vitrectomy combined with glaucoma drainage valve implantation and phacoemulsification cataract extraction. The uncorrected visual acuity (UCVA), intraocular pressure (IOP), and iris neovascularization (INV) scores were recorded and compared among the 3 groups before and after operation, and then the postoperative pain relief and complications were observed.

**Results:**

Through observation, there was no significant difference in the UCVA, IOP, and INV scores in the 3 groups before operation. After the operation, the UCVA, IOP, and INV scores of the 3 groups were significantly lower than those before operation. After operation, the UCVA of the 3 groups increased first and then decreased, and it improved most significantly in the 3rd month after operation and decreased in the 4th month after operation. There were significant differences in UCVA among the 3 groups at each time point after operation. From the 1st day to the 6th month after operation, the IOP of the 3 groups showed an upward trend, and there was no significant difference among the 3 groups in IOP at each time point after operation. At the 1st, 3rd, and 6th months after operation, the INV score of group A and group B was higher than that of group C. There was no significant difference in the INV score between group A and group B. The incidence of complications was not significantly different among the 3 groups.

**Conclusion:**

23G minimally invasive vitrectomy, glaucoma drainage valve implantation, and phacoemulsification cataract extraction can effectively improve the UCVA, IOP, and INV scores of NVG secondary to PDR with VH, and the combined application of the 3 methods has better security.

## 1. Introduction

Diabetes is a metabolic disease, which is mainly manifested as hyperglycemia [1]. Long-term hyperglycemia can lead to different degrees of tissue damage, resulting in dysfunction of the eye, kidney, heart, blood vessels, nerves, and so on [2]. Diabetic retinopathy is a common blinding disease. In the course of disease development, 62% of patients with diabetes can develop iris neovascularization (INV), and 41.4% eventually develop into neovascular glaucoma (NVG); therefore, proliferative diabetic retinopathy (PDR) is the most important stage of evolution to NVG [3]. In a few patients, since diabetic retinopathy (DR) was not found early or treatment was delayed, NVG was diagnosed at the time of treatment. So the intraocular pressure (IOP) of these patients was still higher than 21 mmHg after symptomatic administration with the largest amount of IOP-lowering drugs. In order to eliminate INV and/or angle neovascularization (ANV), antiglaucoma surgery should be performed in time to reduce IOP and protect the residual visual function of NVG patients. NVG secondary to PDR with vitreous hemorrhage (VH) is a common refractory glaucoma case. Ocular pain, photophobia, corneal edema, conjunctival congestion, and poor vision are the main manifestations of the disease. With the incidence rate of diabetes increasing year by year, the incidence rate of NVG also showed an obvious increasing trend [4]. In recent years, a few attempts have been made to treat the infantile cataract by crystalline resection using the minimally invasive vitrectomy [5]. It has been reported that simultaneous vitrectomy and AGV implantation in patients with posterior segment disease-related glaucoma may be an effective option to manage complex glaucoma cases [6]. At present, surgical treatment is the most commonly used treatment for this disease, and 23G minimally invasive vitrectomy, glaucoma drainage valve implantation, and phacoemulsification cataract extraction are commonly used. However, due to the different complexity of the disease, only one surgical method is often unable to meet the requirements of treatment. It has been reported that the treatment of NVG secondary to PDR with VH by multiple surgical methods can better treat the disease [7]. In order to improve the success rate of surgery and improve the condition of patients more effectively, the above three surgical methods are combined for treatment.

## 2. Patients and Methods

### 2.1. Clinical Data

Eighty-three patients (91 eyes) with PDR diagnosed as NVG phase III complicated with VH from June 2018 to May 2020 were selected as the study subjects. The subjects were randomly divided into 3 groups: there were 28 patients (30 eyes) in group A, 27 patients (30 eyes) in group B, and 28 patients (31 eyes) in group C. This study obtained approval from the Ethics Committee of Xiamen University, following the principle of the Declaration of Helsinki (as revised in 2013). The patients have signed the informed consent forms.

The clinical stage of NVG was as follows [8]: phase I (preglaucoma): the iris or anterior chamber angle neovascularization is found; however, as the function of the atrium angle has not been endangered, the IOP is normal, and the patient may have no symptoms; phase II (open-angle glaucoma): the angle of the atrium was not closed, but the neovascular membrane extended into the trabecular meshwork; the function of the trabecular meshwork was damaged, the outflow of aqueous humor was blocked, and the IOP was increased; and phase III (angle-closure glaucoma): the neovascularization membrane contracted, the angle of the atrium adhered and closed, and the IOP increased sharply.

Inclusion criteria were as follows: (1) the age of the patients was more than 18 years old, the patient's disease was nonabsorbable VH caused by PDR, there was obvious INV, and NVG met the criteria of clinical stage III; (2) IOP was still higher than 21 mmHg after topical and systemic administration of the largest dose of IOP-lowering drugs; (3) the results of gonioscopy or ultrasound biomicroscopy showed that the angle was closed in the range of more than 180 degrees; (4) the fasting blood glucose was below 8 mmol/ml, and HbA1c was less than 8.0%; and (5) no treatment was performed 1 month before admission.

Exclusion criteria were as follows: (1) less than 18 years old; (2) history of ocular trauma; (3) history of strabismus surgery, external retinal detachment reattachment, and other conjunctival surgery or PPV surgery; (4) serious corneal edema or bulla formation and unseen fundus; (5) no light perception; (6) obvious lens turbidity and obvious vitreoretinal proliferation or retinal detachment showed by B-ultrasound; (7) patients with coagulation dysfunction and serious organic diseases such as renal insufficiency and cardiac insufficiency who cannot tolerate surgery; and (8) patients with incomplete clinical data or unwilling to participate in this clinical trial.

Experimental grouping was as follows: in group A, there were 15 males (16 eyes) and 13 females (14 eyes), the average age was 56.7 ± 21.1 years (range, 41-77 years), the course of diabetes was 2-6 years, and the average duration was 3.8 ± 2.7 years; in group B, there were 14 males (16 eyes) and 13 females (14 eyes), the average age was 56.9 ± 22.5 years (range, 41-78 years), the course of diabetes was 2-6 years, and the average duration was 3.7 ± 2.6 years; and in group C, there were 14 males (16 eyes) and 14 females (15 eyes), the average age was 58.0 ± 21.7 years (range, 40-79 years), the course of diabetes was 2-6 years, and the average duration was 3.6 ± 2.5 years.

### 2.2. Therapeutic Methods

Before operation, routine examinations such as blood routine examination, urine routine examination, liver and kidney function examination, and electrocardiogram examination were carried out for the three groups of patients to understand the general situation and reduce the risk of surgical emergencies. At the same time, another auxiliary specialist examination was carried out, where the patients were given ophthalmic examination; the best-corrected visual acuity (BCVA) and uncorrected visual acuity (UCVA) were examined by the international standard visual acuity chart; the noncontact tonometer (NCT) and Goldmann applanation tonometer (GAT) were used to measure IOP [9]; the cornea, INV, anterior chamber depth, and lens were examined by the slit lamp microscope; the anterior segment was photographed; fundus examination was performed by the direct ophthalmoscope and anterior ophthalmoscope; B-ultrasound was used to examine the vitreous body and retina; gonioscopy was used to examine INV and angle closure. There was no significant difference in gender, age, IOP, and BCVA among the 3 groups (*P* > 0.05, Table 1).

### 2.3. The Method of Intravitreal Injection [10]

Three groups of patients were given topical anesthesia; the eyes were routinely disinfected and covered with a sterile towel; then, the operation was completed by the same surgeon. A 4.5 needle was inserted into the center of the vitreous cavity at 4 mm behind the subtemporal cornea perpendicular to the eye wall; after a slow injection of 0.05 ml (0.5 mg) of conbercept, the needle was withdrawn slowly and then covered with sterile gauze and dropped with ofloxacin eye drops.

### 2.4. 23G Minimally Invasive Vitrectomy [11]

Local anesthesia and disinfection were performed on the patients, and 23G minimally invasive vitrectomy was performed in the flat area of the ciliary body. Three standard incisions were used to peel off the fibrous vascular membrane of the fundus, regulate hemostasis by underwater electrocoagulation, preserve the anterior capsule of the lens, and take out the epithelial cells of the anterior capsule and polish it. Then, cut the vitreous body, completely cut the preretinal fibroproliferative membrane with a 23G cutting head, then perform extensive retinal photocoagulation and silicone oil tamponade, and finally pull out the cutting sleeve.

### 2.5. Glaucoma Drainage Valve Implantation [12]

Cut the bulbar conjunctiva and fascia of the superior temporal quadrant at 0.50 cm from the membranous margin of the cornea, separate the sclera at an angle of about 85 degrees, and infiltrate the local fascia with 5-fluorouracil for 3 min and then wash with normal saline. Perform suture ligation on the root of the adjusted Ahmed glaucoma drainage device, and use the nonabsorbable suture 5-0 to fix the drainage disc 0.80 cm behind the corneal limbus. At the same time, make a scleral tunnel at 0.25 cm behind the limbus, inject the viscoelastic material in the front at 9 o'clock, insert the drainage tube 0.20 cm away from the anterior chamber, and fix the drainage valve with nylon thread at last.

### 2.6. Phacoemulsification Cataract Extraction [13]

After the scleral tunnel was established, perform continuous curvilinear capsulorhexis according to the procedure of phacoemulsification. For sufficient subcapsular separation, in other words, inject the perfusate under the anterior capsule membrane with a blunt needle to separate the lens capsule from the subcapsular cortex. The lens nucleus was emulsified by capsule plane segmentation to absorb the residual cortex. Appropriately expand and place the incision according to the size of the intraocular lens in the capsule bag. Then, suture the fascia and conjunctiva, which can lead to postoperative routine anti-infection, bandaging, and hemostasis.

Group A was treated with 23G minimally invasive vitrectomy combined with glaucoma drainage valve implantation. Group B was given 23G minimally invasive vitrectomy combined with phacoemulsification cataract extraction. Group C was treated with 23G minimally invasive vitrectomy combined with glaucoma drainage valve implantation and phacoemulsification cataract extraction. The operation methods of the 3 groups were the same as above.

### 2.7. Observation Index

Record the UCVA (Log MAR) before operation and at the 1st-6th months after operation. In the absence of antiglaucoma drugs, measure the IOP of the 3 groups by the Schiotz indentation tonometer, and take the mean value of 3 measurements during the above periods. INV was scored according to the Teich and Walsh INV scoring standards, also in the same time period above. The relief of eye pain and complications such as inflammatory exudation of the anterior chamber, anterior chamber hemorrhage, corneal edema, and vitreous rebleeding were observed in the three groups.

### 2.8. INV Grading Standards [14]

No INV was defined as grade 0 (0 points). The presence of INV in 1-2 quadrants was defined as grade 1 (1 point). The presence of INV in 3-4 quadrants was defined as grade 2 (2 points). The presence of INV with the infiltrating matrix in 1-2 quadrants was defined as grade 3 (3 points). The presence of INV with the infiltrating matrix in 3-4 quadrants was defined as grade 4 (4 points). On the basis of grade 4, combined with INV, glaucoma was defined as grade 5 (5 points).

### 2.9. Statistical Analysis

SPSS 23.0 software (IBM Corp.) was used for the statistical analysis of the data. The measurement data were expressed as $\bar{x}\pm s$. The *F*-test was used for multigroup comparison, and repeated measurement ANOVA was used for comparison at different time points. The count data were expressed as cases (%), and the comparison was made by the chi-squared test. The difference was statistically significant when *P* < 0.05.

## 3. Results

### 3.1. Results of UCVA

Before operation, there was no significant difference in the UCVA among the 3 groups (*P* > 0.05). After operation, the UCVA of the 3 groups increased first and then decreased, and it improved most significantly in the 3rd month after operation and decreased in the 4th month after operation. There were significant differences in UCVA among the 3 groups at each time point after operation (*P* < 0.05). In the 1st month after operation, the UCVA scores of the 3 groups were in the order of group A, group C, and group B from small to large. From the 2nd month to the 6th month, the UCVA scores of the 3 groups were in the order of group C, group A, and group B from small to large. The results are shown in Figure 1.

### 3.2. Results of IOP

Before operation, there was no significant difference in the IOP among the 3 groups (*P* > 0.05). From the 1st day to the 6th month after operation, the IOP of the 3 groups was significantly lower than that before operation (*P* < 0.05). From the 1st day to the 6th month after operation, the IOP of the 3 groups showed an upward trend, and there was no significant difference among the 3 groups in IOP at each time point after operation (*P* > 0.05). The results are shown in Figure 2.

### 3.3. Results of the INV Score

Before operation, there was no significant difference in the INV score among the 3 groups (*P* > 0.05). At the 1st, 3rd, and 6th months after operation, the INV score of the 3 groups was significantly lower than that before operation (*P* < 0.05). The INV score of group A and group B was higher than that of group C (*P* < 0.05). There was no significant difference in the INV score between group A and group B (*P* > 0.05). The results are shown in Table 2.

### 3.4. Results of Postoperative Pain Relief and Complications

Three days after operation, no obvious eye pain was found in all 3 groups, and the clinical symptoms were relieved. Postoperative complications such as anterior chamber inflammatory exudation, anterior chamber hemorrhage, corneal edema, and vitreous rebleeding occurred in all 3 groups. The incidence rate of complications in group A, group B, and group C was 23.3%, 20.0%, and 25.8%, and there was no significant difference among the 3 groups (*χ*^2^ = 0.315, *P* > 0.05). The results are shown in Table 3.

### 3.5. Typical Cases

Figures 3–6 show the comparison of the same patient before and after operation. The patient is a 68-year-old male with a 10-year history of diabetes, and he uses insulin to control his blood sugar, but his blood sugar is not well controlled. The patient's visual acuity decreased for 1 year, with severe pain in the right eye accompanied by headaches for 4 days. The specialist examination results were as follows: the visual acuity of the right eye includes light perception, conjunctival hyperemia, corneal haze edema, mydriasis, and disappearance of light reflection. The depth of the anterior chamber was normal, a large number of new blood vessels were seen in the iris, the lens opacity was (+ +), and the fundus was not clear. The results of ocular ultrasound were as follows: DR and VH in the right eye. Then, he was treated with 23G minimally invasive vitrectomy combined with glaucoma drainage valve implantation and phacoemulsification cataract extraction. One week after operation, the regression of INV could be observed.

## 4. Discussion

The main cause of PDR complicated with NVG is retinal ischemia or hypoxia caused by central retinal vein occlusion and diabetic retinopathy, which eventually leads to refractory glaucoma. The pathogenesis is the release of the vascular endothelial growth factor (VEGF), platelet-derived growth factor (PDGF), and basic fibroblast growth factor (bFGF) from the ischemic retina and damaged vascular wall to the adjacent retinal tissue, deep choroid tissue, and vitreous cavity; these angiogenesis-promoting factors specifically act on the receptors of vascular endothelial cells and promote the mitosis of vascular endothelial cells; when the adjacent retinal neovascularization proliferates, the remaining proliferative factors diffuse into the vitreous body and enter the posterior chamber, then, with the circulation of aqueous humor through the posterior chamber and anterior chamber, it reaches the angle of the atrium, causing the formation of neovascularization in these parts [15]. Neovascular glaucoma with vitreous hemorrhage is not only complicated in the local eye but also difficult to establish an effective filtering channel through filtering surgery. At present, the treatment of neovascular glaucoma includes the following: the treatment of primary disease, the elimination of the retinal ischemic state (panretinal photocoagulation), and the drug or surgical control of IOP. The main surgical methods include filtration surgery, aqueous humor drainage implantation, and ciliary body destruction surgery [16]. Because the neovascularized fibrous membrane can cause extensive peripheral anterior synechia and destroy the anatomic structure of the angle of the anterior chamber, it is difficult to cut the iris root, easily injure the ciliary body, and cause serious bleeding, so anterior chamber hemorrhage is a common complication after operation [17]. In addition, because of intraoperative and postoperative bleeding, fibrin exudates and blocks the filtering mouth, resulting in adhesion and atresia; the filtration operation is difficult to work. However, because of the difficult curative effect and serious complications, all kinds of ciliary body destructive surgery are not usually chosen by clinicians. Therefore, we use glaucoma decompression valve drainage implant surgery, greatly improving the success rate of surgery.

The principle of the glaucoma decompression valve is to increase the formation of functional filtering blebs by means of a drainage disc on the surface of the sclera. The decrease of IOP depends on the drainage of aqueous humor around the drainage disc. Aqueous humor passively diffuses or penetrates into the intercellular space of orbital tissue and is absorbed by capillaries or lymphatic vessels, resulting in the decrease of IOP [18]. The thinner the wrapping wall, the lower the IOP, and the larger the surface area of the package, the lower the IOP. The Ahmed glaucoma valve is designed as a drainage disc with a large surface area to enlarge the area of scleral surface wrapping. The second is to provide a one-way pressure-sensitive valve to limit the outflow resistance of aqueous humor, which can prevent excessive drainage of aqueous humor before the surface of the drainage disc is wrapped, which can play a long-term role in controlling IOP [19]. In this study, vitrectomy should be combined with other methods because of vitreous hemorrhage. The purpose of vitrectomy is to remove the turbid vitreous hemorrhage, find out the causes of vitreous hemorrhage, and prevent the occurrence of hemocytosis or hemolytic glaucoma. After vitrectomy, the vitreous cavity becomes a liquid cavity, which provides the conditions for the implantation of the aqueous humor drainage tube through the pars plana of the ciliary body, which is more important for those patients who cannot be implanted with the aqueous humor drainage tube through the anterior chamber. Phacoemulsification is to smash the nucleus of the lens into a chylous shape and then suck it out together with the cortex. It can keep the posterior capsule of the lens, which is conducive to the implantation of the posterior chamber intraocular lens.

All patients were given the conbercept injection before operation. Conbercept is a commonly used antivascular endothelial growth factor drug in the clinic. It has high bioavailability and can penetrate the retina well, inhibit the binding of the vascular endothelial growth factor and receptor and neovascularization, and reduce the permeability of new blood vessels, which is conducive to follow-up surgical treatment [20]. The results of this study show that the UCVA, IOP, and INV scores of the 3 groups significantly improved after operation; the reason may be that the neovascularization of the iris and retina can be controlled by conbercept before operation. Vitrectomy can relieve vitreoretinal traction, peel off the fibrovascular membrane and proliferative membrane, remove vitreous hemorrhage, and inhibit neovascularization in PDR eyes to a certain extent. In glaucoma drainage valve implantation, the drainage valve was installed in the corresponding position of the anterior chamber or vitreous cavity and conjunctiva to fascia so as to inhibit neovascularization and reduce IOP by establishing an outflow channel of aqueous humor. Phacoemulsification can remove the turbid lens and put in the intraocular lens; the angle of the anterior chamber is wider than that of the anterior chamber, which is beneficial for the posterior aqueous humor to enter the anterior chamber, reduce the IOP, and further inhibit the formation of neovascularization [21]. In this study, all the 3 groups had postoperative complications, but there was no significant difference in the incidence of complications among the 3 groups, suggesting that the combination of multiple methods for the treatment of NVG with PDR and VH is safe; this may be due to the 3 surgical methods causing less eye irritation, hence fewer complications.

## 5. Conclusion

23G minimally invasive vitrectomy can be combined with glaucoma drainage valve implantation and phacoemulsification cataract extraction. The combination of the 3 methods can effectively improve the UCVA, IOP, and INV scores of PDR patients diagnosed as NVG complicated with VH. In addition, the combined application of the 3 methods is more effective than that of the two methods, and the combined application of the 3 methods has better security. Therefore, the combination of the above 3 methods in the treatment of NVG with PDR and VH is worthy of clinical promotion.

## Figures and Tables

**Figure 1:** Comparison of UCVA among the 3 groups.

**Figure 2:** Comparison of IOP among the 3 groups.

**Figure 3:** Photograph of the right eye of a patient before operation.

**Figure 4:** Enlarged photograph of iris neovascularization.

**Figure 5:** Ultrasound picture of vitreous hemorrhage before operation.

**Figure 6:** Photograph of the right eye of a patient after operation.

**Table 1:** Comparison of baseline data among the 3 groups.

Group	Number of eyes	Sex (male/female, number of cases)	Age ($\bar{x}\pm s$, year)	IOP ($\bar{x}\pm s$, mmHg)	BCVA (number of eyes)					
					NLP	LP	HM	CF/BE	0.01-0.1	≥0.1
Group A	30	15/13	56.7 ± 21.1	49.25 ± 9.73	4	2	9	2	11	2
Group B	30	14/13	56.9 ± 22.5	52.07 ± 10.33	3	2	11	2	9	3
Group C	31	14/14	58.0 ± 21.7	48.65 ± 11.79	4	3	8	4	8	4
*P*		0.910	0.639	0.704	0.301					

**Table 2:** Comparison of the INV score among the 3 groups ($\bar{x}\pm s$, point).

Group	Number of eyes	Before operation	1st month after operation	3rd month after operation	6th month after operation
Group A	30	4.47 ± 0.36	3.07 ± 0.62^∗^^#^	2.06 ± 0.39^∗^^#^	1.83 ± 0.41^∗^^#^
Group B	30	4.51 ± 0.31	2.95 ± 0.57^∗^^#^	2.04 ± 0.28^∗^^#^	1.77 ± 0.24^∗^^#^
Group C	31	4.55 ± 0.29	2.04 ± 0.33^∗^	1.26 ± 0.22^∗^	0.82 ± 0.30^∗^

Note: ^∗^ means compared with the data before operation in the same group, *P* < 0.05; ^#^ means compared with group C, *P* < 0.05.

**Table 3:** Comparison of postoperative complications among the 3 groups (number of eyes/%).

Group	Number of eyes	Anterior chamber inflammatory exudation	Anterior chamber hemorrhage	Corneal edema	Vitreous rebleeding occurred	Incidence rate (%)
Group A	30	2	3	1	2	23.3%
Group B	30	1	2	2	1	20.0%
Group C	31	3	2	1	2	25.8%

## Data Availability

The datasets used and/or analyzed during the current study are available from the corresponding author on reasonable request.
